# COMP-Angiopoietin-1 Recovers Molecular Biomarkers of Neuropathy and Improves Vascularisation in Sciatic Nerve of ob/ob Mice

**DOI:** 10.1371/journal.pone.0032881

**Published:** 2012-03-06

**Authors:** Joanna Kosacka, Marcin Nowicki, Nora Klöting, Matthias Kern, Michael Stumvoll, Ingo Bechmann, Heike Serke, Matthias Blüher

**Affiliations:** 1 Department of Medicine, University of Leipzig, Leipzig, Germany; 2 Institute of Anatomy, University of Leipzig, Leipzig, Germany; 3 IFB Adiposity Disease, University of Leipzig, Leipzig, Germany; Julius-Maximilians-Universität Würzburg, Germany

## Abstract

**Background:**

Leptin-deficient *ob/ob* mice are a model of type 2 diabetes induced peripheral neuropathy. *Ob/ob* mice exhibit obesity, insulin resistance, hyperglycaemia, and alterations of peripheral nerve fibres and endoneural microvessels. Here we test the hypothesis that cartilage oligomeric matrix protein (COMP)-Ang-1, a soluble and stabile form of Ang-1 which promotes angiogenesis and nerve growth, improves regeneration of nerve fibres and endoneural microvessels in *ob/ob* mice.

**Methods and Findings:**

COMP-Ang-1 (100 ng/ml) or NaCl were intraperitoneally (i.p.) injected into male (N = 184), 3-month old, *ob/ob* or *ob/+* mice for 7 and 21 days. We measured expression of Nf68, GAP43, Cx32, Cx26, Cx43, and TNFα in sciatic nerves using Western blot analysis. To investigate the inflammation in sciatic nerves, numbers of macrophages and T-cells were counted after immunofluorescence staining. In ultrathin section, number of myelinated/non-mylinated nerve fibers, g-ratio, the thickness of Schwann cell basal lamina and microvessel endothelium were investigated.

Endoneural microvessels were reconstructed with intracardial FITC injection. Treatment with COMP-Ang-1 over 21 days significantly reduced fasting blood glucose and plasma cholesterol concentrations compared to saline treated *ob/ob* mice. In addition, COMP-Ang-1 treatment: 1) up-regulated expression of Nf68 and GAP43; 2) improved expression of gap junction proteins including connexin 32 and 26; 3) suppressed the expression of TNFα and Cx43 and 4) led to decreased macrophage and T-cell infiltration in sciatic nerve of *ob/ob* mice. The significant changes of sciatic nerve ultrastructure were not observed after 21-day long COMP-Ang-1 treatment. COMP-Ang-1 treated *ob/ob* mice displayed regeneration of small-diameter endoneural microvessels. Effects of COMP-Ang-1 corresponded to increased phosphorylation of Akt and p38 MAPK upon Tie-2 receptor.

**Conclusions:**

COMP-Ang-1 recovers molecular biomarkers of neuropathy, promotes angiogenesis and suppresses inflammation in sciatic nerves of *ob/ob* mice suggesting COMP-Ang-1 as novel treatment option to improve morphologic and protein expression changes associated with diabetic neuropathy.

## Introduction

Peripheral diabetic neuropathy (PDN) is a serious complication of diabetes which is associated with neurotrophic changes, demyelination and degeneration of all fiber types, loss of sensory fibers, alterations of endoneural microvessels and decreased performance of the perineurium blood-nerve barrier in the peripheral nerve [1], [2], [3], [4]. Increasing evidence suggests that the pathogenesis of diabetic neuropathy is multifactorial [5]. Chronic hyperglycaemia, increased levels of advanced glycation end products (AGEs), reactive oxygen species (ROS) and inflammatory cytokines significantly contribute to the development of PDN [5], [6], [7]. Until now, there is no causal treatment of diabetic neuropathy and improvement of glycaemic control is the only way to minimize the risk of PDN [8].

Leptin-deficient *ob/ob* mice are widely accepted as an animal model of type-2 diabetes induced PDN [9]. Drel and co-authors [9] demonstrated that *ob/ob* mice have motor and sensory nerve conduction deficits, small sensory nerve fiber neuropathy, intraepidermal sensory nerve fiber loss as well as oxidative-nitrosative stress in peripheral nerve, spinal cord, and dorsal root ganglions (DRG). These alterations of the peripheral nervous system are most likely related to the phenotype of *ob/ob* mice, which exhibit over 50% body fat mass, insulin resistance, hyperglycaemia and alterations of endoneural microvessels [10], [11].

Angiopoetin-1 has been shown to act anti-apoptotic and neurotrophic on neurons of central – and peripheral nervous system *in vitro* [12], [13], [14], [15]. Recently, cartilage oligomeric matrix protein (COMP) -angiopoietin-1 (Ang-1) has been developed as a soluble, stable, and potent Ang-1 variant which was shown to protected against radiation-induced apoptosis in microcapillary endothelial cells of the intestinal villi and prolonged survival [16]. Recombinant COMP-Ang-1 was generated by replacing the N-terminal portion of Ang-1 with the short coiled-coil domain of cartilage oligomeric matrix protein, which is more potent than native Ang-1 in phosphorylation of Tie-2 receptor [16]. The Ang-1/Tie-2 system is involved in endothelial cell migration, pericyte recruitment as well as formation, remodelling and maturation of blood vessels [17], [18] and promotes angiogenesis and neuritogenesis, thereby coordinating the healing process of injured nerve fibres and endoneural microvessels [13].

Interestingly, hyperglycemia causes significant reduction of Ang-1 and Tie-2 expression and disruption of Ang-1/Tie-2 signalling pathway [19], [20]. COMP-Ang-1 was further shown to activate osteogenesis by promoting angiogenesis in spinal fusions [21], decreases lipopolysaccharide-and ischemia reperfusion induced acute kidney injury [22]. Based on the beneficial effects of COMP-Ang-1 on angiogenesis and nerve growth, we here test the hypothesis that COMP-Ang-1 may improve regeneration of nerve fibres and endoneural microvessels in *ob/ob* mice.

## Materials and Methods

### Animals

Male (N = 184; Table 1), 3-month old, *ob/ob* homozygote and *ob/+* heterozygote (B6.V-Lep ^ob/ob^ and B6.V-Lep ^ob/J^) mice were obtained from the Taconic Europe (Ry, Denmark) and body weight was recorded for each group (*ob/+*: mean 27 g, range 26–28 g; and *ob/ob*: mean 48 g, range 47–49 g). Mice were adjusted to the local animal facilities (3–6 mice per group and cage) and maintained at 21±1°C on a 12 h light/dark cycle; mice had free access to water and were fed with regular food (Global Rodent T.2018.R12 from Harlan Teklad, containing 12% of calories from fat). Experiments followed the international guidelines for the prevention of animal cruelty and were approved by the Regierungspräsidium Leipzig, the local authority for animal care (TVV 11/10). All mice were sacrificed via a CO_2_ overdose. The sciatic nerves were dissected and the number of endoneural microvessels, expression of structural and proinflammatory proteins as well as crucial signaling pathways were evaluated.

**Table 1:** The number of animals used in experiments. The experimental groups: NaCl ob/+, NaCl ob/ob, COMP‐Ang‐1 ob/+ and COMP‐Ang‐1 ob/ob mice.

	7 days of treatment	21 days of treatment	total number
	n (per each group)	n (per each group)	
Western blot**:**			
Nf68, GAP43	4	4*	32
Cx32, Cx26	4	4*	32
TNFα, Cx43	4	4	32
Ang-1, Tie-2, p-Tie-2		4	16
Akt,p-Akt, p38 MAPK, p-p38 MAPK		4	16
reconstruction of endoneural Microvessels		6°	24
Immunostaining: Iba1, CD3, TNFα Nf200		5	20
transmission electron microscopy		3	12
			**184**

* lipid status

°blood glucose concentrations and body weight

### Application of COMP-Ang-1

COMP-Ang-1 (Axxora Deutschland GmbH, Lörrach, Germany; 100 ng/ml, diluted in sterile 0.9% NaCl) or sterile 0.9% NaCl solution (B. Braun, Melsungen, Germany; 5 µl/1 g body weight) were intraperitoneally (i.p.) injected into *ob/ob* or *ob/+* mice every 24 h, for 7 or 21 days. A fasting whole-blood glucose concentration ≥16 mmol/l in *ob/ob* mice and 5–8 mmol/l in *ob/+* control mice were the criteria to include the animals in the intervention studies.

### Lipid status and blood glucose concentration

Blood glucose concentration was measured using an Opticum Omega glucometer (GlucoMen, Menarini Diagnostics, Berlin, Germany) in whole blood taken from the ventral caudal vein at baseline, 1, 4, 7, 14 and 21 days after COMP-Ang-1 or NaCl injection

Blood samples (0.5 ml) for lipid status were taken by cardiac puncture between 8 and 10 AM, 21 days after administration of the COMP-Ang-1 or NaCl. Triglyceride, HDL/LDL cholesterol were determined in the supernatant (ELISA; Linco, St. Charles, USA) (n = 6 per group).

### Immunoblotting

Sciatic nerves of each group (n = 4) were lysed by ultrasonication in 60 mM Tris-HCl, pH 6.8, containing 2% sodium dodecyl sulfate (SDS) and 10% sucrose. Tissue lysates were diluted 1∶1 in sample buffer (250 mM Tris-HCl, pH 6.8, containing 4% SDS, 10% glycerol, and 2% b-mercaptoethanol) and denatured at 95°C for 5 min. Protein concentration was assessed with the BCA protein assay (Pierbo Science, Bonn, Germany). Proteins (30 µg per lane) were separated by electrophoresis on a 12.5% or 15% SDS-polyacrylamide gel and transferred to nitrocellulose by electroblotting. Nonspecific binding sites were blocked with 5% dry milk for 45 min, then subsequently incubated with primary antibodies: mouse anti-neurofilament 68 (NF68, clone NR4), mouse anti-growth associated protein (GAP) 43 (Sigma Aldrich; Taufkirchen, Germany, 1∶2 000) rabbit anti-Connexin (Cx) 26, mouse anti-Cx32 (Millipore, Schwalbach, Germany), mouse anti-Cx43 (Clone CXN-6; Sigma), tumour necrosis factor alpha (TNFα, Abcam, MA, USA; 1∶1 000), goat anti-Ang-1 (Santa Cruz Biotechnology, Santa Cruz, CA; 1∶500), anti-mouse Tie-2, rabbit anti-phospho-Tie-2 (all from R&D Systems, Wiesbaden-Nordenstadt, Germany; 1∶2 000), rabbit Akt, phospho-Akt (Ser473) mouse mAb, rabbit p38MAPK, phospho-p38MAPK (Thr180/Tyr182) mouse mAb (all from Millipore; 1∶1 000) at 4°C overnight. Proteins were detected by incubating with HRP conjugated secondary antibodies at a 1∶3 000 dilution; Dianova) at RT for 2 h and chemiluminescence kit (Amersham, Pharmacia, Freiburg, Germany). Integrated optical densities of the immunoreactive protein bands were measured with Gel Analyzer software (Media Cyberneties, Silver Spring, MD). Equal protein loading was verified using mouse anti-D-glyceraldehyde-3-phosphate dehydrogenase antibody (GAPDH, Research Diagnostics, Flanders, The Netherlands; 1∶3 000).

### Immunostaining

Mice (n = 5 per group) were perfused with 4% paraformaldehyde in 0.1 M PBS. Dissected sciatic nerves were postfixed in the same fixative for 4 hr, rinsed with PBS, transferred into 30% buffered sucrose solution, and stored at 4°C until sectioning. The 10-µm-thick frozen cross sections were mounted on gelatinized glass slides. After buffer rinse, sections were incubated with rabbit polyclonal microglia/macrophage cytoplasmatic calcium adaptor Iba-1 antibody for the detection of macrophages (1∶200; WAKO Chemicals USA, Richmond, VA) or with rabbit polyclonal CD3 for detection of T-cells (1∶200; Dako Cytomation, Hamburg, Germany) in double staining with the mouse monoclonal antibody against neurofilament 200 (NF200; 1∶500; Sigma Aldrich, Taufkirchen, Germany). For co-localization study, Iba-1 and CD3 antibody was used in combination with the mouse monoclonal TNFα antibody (1∶100; Abcam, ab1793) at 4°C overnight. After buffer rinse, Cy3-conjugated goat anti-mouse IgG (Dianova) with FITC-conjugated goat anti-rabbit IgG was diluted 1∶700, and sections were incubated at room temperature for another 2 h. Sections were mounted with Dako Glycergel (Dako Cytomation) containing 10 µg/ml DAPI (Serva, Heidelberg, Germany) for nuclear staining and 25 µg/ml DABCO (Sigma) to prevent photobleaching. By replacement of the primary antisera with normal mouse IgG, rabbit serum or PBS, respectively, no specific immunoreaction occurred.

### Determination of macrophages and T-cells

Digitalized pictures were taken with the LSM 510 Meta confocal microscope (Zeiss). The number of macrophages and T-cells was counted in cross sciatic nerve sections (n = 5, in each experimental group) stained by immunohistochemistry for Iba-I (a macrophage marker) or CD3 (a T cell marker). Values represent numbers of stained cells per mm^2^.

### Endoneural microvessel detection by fluorescein isothiocyanate-dextran (FITC)

Immediately upon death, each animal (n = 6 per group) were perfused via the left heart ventricle, first with 5 ml phosphate buffered saline (PBS, pH 7.4) containing 6250 u/l heparin (Sigma, Taufkirchen, Germany), and then 5 ml 4% formaldehyde in PBS, followed by 10 mg/ml FITC (Sigma) in PBS. All perfusion buffers were warmed to 37°C. Sciatic nerves from both the right and left side dissected above division into fibular and tibial nerve were mounted on a cork-plate, postfixed in 4% buffered formaldehyde for 1 h, rinsed with PBS, and embedded on glass slides with Glycergel mounting medium (DAKO Cytomation, Hamburg, Germany).

### Transmission electron microscopy

The left sciatic nerves of each group (n = 3) were fixed in 2% glutaraldehyde with 1% paraformaldehyde in 0.1 M PBS at 4°C for 2 h, and postfixed in 1% buffered osmium tetroxide (1.5 h, 4°C). Cross-cut samples of the sciatic nerves were transferred into 70% acetone, treated with 1% phosphotungstic acid and 1% uranyl acetate (20°C, 1 h) and further dehydrated in acetone. Samples were embedded in resin (Durcopan® ACM Fluka, Sigma-Aldrich, Steinheim Germany) and polymerized at 60°C for 48 h. Semithin sections were stained with 1% toluidine blue solution; ultrathin sections were mounted on copper grids, contrasted with uranyl acetate and lead citrate, and analyzed using an EM 900 electron microscope (Zeiss, Jena, Germany).

### Thickness of myelin sheath and number of myelinated/non-mylinated nerve fibers

To measure the thickness of the myelin sheath, digitalized photographs were taken from cross-cut ultrathin sections of two samples per mouse at 3000× magnification. To begin with the upper left corner of the grid, a total of 50 pictures were obtained for each nerve. Nerve fibers of round to oval forms were selected according to Weibel (1963); the smallest diameter was measured for the axon and nerve fiber size by the TRS Docu TEM Package software (Zeiss, Oberkochen, Germany), and the myelin sheath thickness was estimated as a g-ratio (obtained by axon diameter/fiber diameter ratio for each axon). To ensure blinded investigations, measurements were conducted without the knowledge of the genotypes. In addition, the absolute number of non-myelinated and myelinated fibers was assessed per 400 µm^2^ area from 50 pictures for each nerve.

### Thickness of Schwann cell basal lamina

We also measured the thickness of the basal lamina of Schwann cells (approximately 150 cells per nerve from 30 digitalized TEM-pictures; 90% of Schwann cells related to myelinated fibers) using the TRS Docu TEM Package software (Zeiss).

### Thickness of endoneural microvessel endothelium

The smallest diameter was measured for the capillary lumen and capillary by the TRS Docu TEM Package software (Zeiss). Thickness of endoneural microvessel endothelium was validated as a capillary lumen diameter/capillary diameter ratio.

### Statistical analyses

Data are presented as means ± SEM or ± SD. Differences among the groups were validated by one-way-ANOVA and the Newman-Keuls test using SigmaStat (Jandel Scientific, San Rafael, CA). A value of p<0.05 was considered statistically significant.

## Results

### COMP-Ang-1 treatment decreases blood glucose and plasma cholesterol concentrations in *ob/ob* mice

The application of COMP-Ang-1 significantly decreased blood glucose concentration in hyperglycaemic ob/ob mice compared with NaCl treated animals. After 21 days treatment, fasting blood glucose concentration of *ob/ob* mice was indistinguishable from non-diabetic *ob/+* controls (Fig. 1A). COMP-Ang-1 had no effect on blood glucose concentration in non-diabetic ob/+ control mice (Fig. 1A).

**Figure 1:** Effect of COMP-Ang-1 treatment on blood glucose concentrations and body weight. Metabolic parameters and body weight of *ob/ob* mice and non-diabetic *ob/+* control mice with COMP-Ang-1 (100 ng/ml) or NaCl treatment. COMP-Ang-1 significantly decreased blood glucose level (A) in ob/ob mice compared with NaCl treatment at 21 days. After 21 days, glucose concentration was indistinguishable between COMP-Ang1 treated *ob/ob* and non-diabetic *ob/+* mice. (B) Effect of COMP-Ang-1 treatment of body weight. Data are means ±SD; n = 6 per group.

HDL- and LDL-cholesterol plasma concentrations were significantly higher in *ob/ob* mice, whereas circulating triglycerides were lower compared to *ob/+* mice (Table 2). Significant decrease about 54% of total cholesterol and about 28% increase of triglyceride serum concentrations were observed in *ob/ob* mice after 21 days of the COMP-Ang-1 treatment (Table 2). Noteworthy, these effects of COMP-Ang-1 treatment were independent of the body weight, which did not significantly change during the study course in *ob/ob* and *ob/+* mice (Fig. 1B). Only saline treated *ob/ob* mice showed a tendency for increased body weight during the last week of treatment (Fig. 1B).

**Table 2:** COMP-Ang-1 treatment (100 ng/ml) effect of ob/ob and ob/+ mice on lipid profile after 21 days.

[mmol/l]	ob/ob		ob/ob		ob/+		ob/+	
	NaCl		COMP-Ang-1		NaCl		COMP-Ang-1	
		±SD		±SD		±SD		±SD
Triglyceride	**0.56**	0.03	**0.78**	0.02	**0.83**	0.01	**0.85**	0.04
Cholesterol	**4.47**	0.67	**2.08**	0.08	**1.71**	0.19	**1.89**	0.22
HDL-Cholesterol	**2.78**	0.45	**1.68**	0.29	**1.47**	0.09	**1.48**	0.13
LDL-Cholesterol	**0.65**	0.16	**0.19**	0.01	**0.15**	0.02	**0.16**	0.02

The COMP-Ang-1 dependent decrease of plasma cholesterol and increase of triglyceride were noted in ob/ob mice. Data are means ± SD; n = 6 per group.

### Effect of COMP-Ang1 treatment on neuron-structural protein expression

Neurofilaments (Nfs) are major determinants of axonal calibre whereas growth associated proteins (GAPs) belong to membrane-associated plasticity markers. Noteworthy, in experimental diabetes and diabetic patients, alterations of peripheral nerve are associated with decreased expression of Nfs and GAPs [3], [23]. Therefore, we tested the effects of COMP-Ang-1 treatment on Nf68 and GAP43 protein expression, both after 7 and 21 days of treatment. In *ob/ob* mice, COMP-Ang-1 application resulted in about 57% and 59% increase of Nf68 protein expression on day 7 and 21 when compared with NaCl treated group (Fig. 2). On day 7, no changes of GAP43 protein levels were noted between COMP-Ang-1 and NaCl treated ob/ob mice. Strikingly, COMP-Ang-1 caused the increase (about 91%) of GAP43 expression in ob/ob mice compared with NaCl treated animals on day 21 of application (Fig. 2).

**Figure 2:** Expression of NF68 and GAP43 in sciatic nerve biopsies of *ob/ob* and *ob/+* mice. (A) Representative Western blots and corresponding densitometrical analyses (B) of neurofilament (NF) 68 and growth associated protein (GAP) 43 in sciatic nerve of *ob/ob* and *ob/+* mice treated with COMP-Ang-1. The decreased level of NF68 protein and strikingly down-regulation of GAP43 indicates on degeneration of nerve fibres in the sciatic nerve of *ob/ob* mice compared with *ob/+* controls. COMP-Ang-1 treatment significantly up-regulates expression of both neural-structural proteins in *ob/ob* mice compared with NaCl treatment at 21 days. (B) Data from n = 4 are presented as mean ±SEM. * p≤0.05, ** p≤0.01, *** p≤0.001, according to the one-way analysis of variance together with the Newman-Keuls test. GAPDH was used as normalization control.

### Effect of COMP-Ang-1 on gap-junction and pro-inflammatory protein expressions in sciatic nerve of *ob/ob* mice

Gap junction proteins - connexins (Cx) are an important component in the maintenance of the perineurium blood-nerve barrier. Several studies have demonstrated that perturbation of this barrier and altered expression of connexins contribute to diabetes related neuropathy [4], [24], [25]. Therefore, the expression of Cx26, 32 and 43 was examined in sciatic nerve of *ob/ob* and *ob/+* mice. In NaCl treated groups, a significant reduction of Cx26 (about 72%) and Cx32 (about 90%) was observed in sciatic nerves of *ob/ob* mice when compared with *ob/+* controls (Fig. 3). In contrast, significantly increased levels of Cx43 (about 50%) were detected in *ob/ob* mice compared with *ob/+* animals (Fig. 3). COMP-Ang-1 treatment resulted in about 50% increase of Cx26 protein expression as well as in about 83% and 92% increase of Cx32 protein level on days 7 and 21, respectively. Cx43 protein expression was about 11% higher on day 7 and it dropped about 43% on day 21 in COMP-Ang-1 treated *ob/ob* mice compared with saline treated mice (Fig. 3).

**Figure 3:** Effect of COMP-Ang-1 on Cx26, Cx32, Cx43 and TNFα expression in sciatic nerves. Diabetic neuropathy is associated with increased expression of tumour necrosis factor alpha (TNFa) and connexin (Cx) 43 and with decreased expression of Cx26 and Cx32 in endo-/perineurium of sciatic nerve in *ob/ob* mice compared with ob/+ controls. COMP-Ang-1 treatment inhibited up-regulation of pro-inflammatory cytokine TNFa and Cx43 and recovered the synthesis of Cx26 and Cx32 in sciatic nerve of ob/ob mice at 7 and 21 days. (A) Representative Western blots; (B) Data of densitometrical analysis after normalization to GAPDH. Results are presented as mean ±SEM. * p≤0.05, ** p≤0.01, *** p≤0.001, according to the one-way analysis of variance together with the Newman-Keuls test (n = 4).

Up-regulation of Cx43 protein was found to occur in parallel with the increased synthesis of pro-inflammatory cytokine-TNFα in macrophages, Schwann cells, and endothelial cells of diabetic nerves [26], [27], [28]. TNFα plays a pivotal role in pain transmission, nerve degeneration and insulin resistance in diabetes related neuropathies [29], [30]. We therefore tested whether COMP-Ang-1 dependent Cx43 decrease corresponds to changes in TNFα expression. TNFα expression was markedly increased (about 72%) in hyperglycaemic *ob/ob* mice as compared with *ob/+* control animals. In *ob/ob* mice, COMP-Ang-1 treatment significantly decreased TNFα protein level on days 7 (about 17%) and 21 (about 51%) as compared with NaCl treated group (Fig. 3).

### Effect of COMP-Ang-1 on local inflammatory response in sciatic nerve of *ob/ob* mice

To further investigate whether COMP-Ang-1 modulates inflammatory processes in sciatic nerve, the immunostaining against microglia/macrophage cytoplasmatic calcium adaptor Iba-1 for macrophages and CD3 for T-cells was performed in COMP-Ang-1 treated *ob/ob* mice compared with saline treated mice or with the *ob/+* control mice at 21 days.

The sciatic nerves of hyperglycemic *ob/ob* mice showed greater infiltration of macrophages compared with normoglycemic *ob/+* mice. Most interestingly, the COMP-Ang-1 treatment decreased about 45% the macrophage number in sciatic nerves of *ob/ob* mice at 21 days (Fig. 4A, B).

**Figure 4:** Analysis of macrophages and T cells distribution in cross sections of sciatic nerves from *ob/ob* and *ob/+* mice under treatment of COMP-Ang-1 at 21 days. Quantification of Iba-1+ macrophages (A) and CD3+ T-cells (C) activation in sciatic nerves (n = 5). B, D: Double immunofluorescence staining against Iba1 (green, macrophages) or CD3 (green, T cells) and neurofilament 200 (red). Immunoreactivity (arrows) for macrophages and T-cells was higher in nerves of non-treated ob/ob mice compared to COMP-Ang-1 treated ob/ob or ob/+ mice. E: Double immunofluorescence staining against Iba1 (green, macrophages) and TNFα (red). Note that TNFα immunoreactivity co-localizes with macrophages (arrows). Cell nuclei were stained with DAPI (blue). Bar represents 100 µm (B, D) and 30 µm (E) respectively. Results are presented as mean ±SEM. * p≤0.05, ** p≤0.01, *** p≤0.001, according to the one-way analysis of variance together with the Newman-Keuls test.

In contrast, the number of infiltrating T-cells in untreated mice was much lower that the number of infiltrating macrophages. T-cell infiltration appeared to be highest in ob/ob mice vs. *ob/+* mice. An about 47% decrease of T-cells was observed in ob/ob mice under COMP-Ang-1 treatment (Fig. 4C, D).

To identify the cell types, which were immunoreactive for proinflammatory cytokine TNFα, double immunofluorescence staining was performed. The TNF IR co-localized with macrophages (Fig. 4E) and partly with T cells.

### COMP-Ang-1 promotes the regeneration of sciatic nerve endoneural microvessels in *ob/ob* mice

The endoneural microvessels abnormalities precede the axonal degeneration in diabetes related neuropathy [31] and vice versa, revascularization precedes regenerating axons [32], [33]. Therefore, the sciatic nerve endoneural blood vessels of COMP-Ang-1 or NaCl treated ob/ob and *ob/+* mice were examined using FITC injection and then classified into three groups according to their diameters (Fig. 5). NaCl treated *ob/ob* mice showed significantly impaired density of microvessels with the smallest diameter (<5 µm) and more with largest (>10 µm) diameter compared with *ob/+* controls. No differences were observed in the number of microvessels with the medium (5–10 µm) diameter between both groups. Interestingly, COMP-Ang-1 significantly enhanced density of endoneural microvessels with smallest diameter in *ob/ob* mice comparing with NaCl treated group on day 21 of application. The numbers of smallest endoneural microvessels between COMP-Ang-1 treated *ob/ob* and *ob/+* mice were similar (Fig. 5).

**Figure 5:** COMP-Ang-1 dependent regeneration of endoneural microvessels in *ob/ob* mice. COMP-Ang-1 treatment enhanced densities of small-diameter endoneural microvessels in ob/ob mice. Endoneural microvessels were visualized by FITC injection (10 mg/ml). To measure the number and diameter of FITC-injected endoneural microvessels, digitalized pictures were taken with the LSM 510 Meta confocal microscope both in the longitudinal and the cross-cut view per nerve (n = 6) (a–d, scale bars: 50 µm). e: Significantly more endoneural microvessels with a smallest diameter (Ø<5 µm) were found in ob/+ controls, whereas *ob/ob* mice showed degeneration of small-diameter microvessels. COMP-Ang-1 treatment enhanced densities of small-diameter endoneural microvessels in *ob/ob* mice compared with NaCl groups after 21 day-long treatment (a, b, e). f, g: COMP-Ang-1 treatment does not affect the number of endoneural microvessels with the medium (Ø = 5–10 µm) and larger diameter (Ø>10 µm) both in ob/ob and ob/+ mice compared to NaCl treatment.

### Sciatic nerve ultrastructure

No significant differences of fiber morphology, including axons diameters and thickness of the myelin sheath, were found in sciatic nerve of COMP-Ang-1 and saline treated *ob/ob* and *ob/+* mice (Fig. 6d). However, the number of non-myelinated nerve fibers appeared to be higher in COMP-Ang-1 vs. saline treated *ob/ob* mice, but these differences were not statistically significant (Fig. 6e).

**Figure 6:** Analysis of sciatic nerve ultrastructure. a–c: Sciatic nerves with endoneural microvessels of NaCl ob/ob, COMP-Ang-1 ob/ob and NaCl ob/+ mice. d–g: The g-ratio (as axon/fiber diameter), number of myelinated/non-mylinated nerve fibers, endoneural microvessel endothelium and SC basal lamina thicknesses were examined by electron microscopy in COPM-Ang-1 or saline treated ob/ob and ob/+ mice (n = 3). d: There are no significant differences in g-ratio in the all groups. e: The number of non-myelinated nerve fibers appears to be low in saline ob/ob mice compared with ob/+ control mice and increased after 21-day long COMP-Ang-1 treatment, these data were not statistically significant. f: The ratio of endoneural microvessels endothelium thickness shows a statistically significant decrease in ob/ob mice vs. ob/+ mice. g: The thickness of Schwann cells basal lamina is increased in the ob/ob mice. The differences between COMP-Ang-1 and saline treated ob/ob mice were not apparent. Results are presented as mean ±SEM. * p≤0.05, ** p≤0.01 according to the one-way analysis of variance together with the Newman-Keuls test.

The characteristic changes of endoneural microvessel, such as a thickened basement membrane and microvessel endothelium, as well as thickened Schwann cell basal lamina were observed in hyperglycemic *ob/ob* mice vs. normoglycemic *ob/+* mice. No differences were found between saline and COMP-Ang-1 treated ob/ob mice (Fig. 6e, f).

### COMP-Ang-1 induces phosphorylation of Tie-2, Akt and p38-MAPK in sciatic nerve of *ob/ob* mice

Diabetic hyperglycaemia causes impairment of Ang-1 and Tie-2 signalling, closely associated with reduced angiogenesis [19]. Therefore, Ang-1 and Tie-2 protein expressions as well as Tie-2 phosphorylation were examined. There was about 45% drop in Ang-1 protein level in sciatic nerve of NaCl treated *ob/ob* mice compared with *ob/+* controls. COMP-Ang-1 led to about 39% increase of Ang-1 expression level in *ob/ob* mice on day 21 of application (Fig. 7). An about 24% decrease of Tie-2 receptor protein level was noted in saline treated *ob/ob* mice compared with *ob/+* controls. Expression of Tie-2 did not change in response to 21-day COMP-Ang-1 treatment (Fig. 7), however, COMP-Ang-1 application induced phosphorylation of Tie-2 (Fig. 7)

**Figure 7:** Ang-1, Tie-2, Akt and p38 MAPK expression in sciatic nerve biopsies of *ob/ob* and *ob/+* mice. Representative Western blots (A) and corresponding densitometrical analyses (B) of Ang-1, Tie-2, Akt and p38 MAPK and in sciatic nerve of *ob/ob* and *ob/+* mice under treatment of COMP-Ang-1. A: COMP-Ang-1 led to the increase of Ang-1 expression in ob/ob mice on day 21 of application and improved the expression of phospho–Tie2, -Akt and -p38 MAPK after 60 min of the injection in both ob/ob and ob/+ mice. B: Results are presented as mean ±SEM. ** p≤0.01, *** p≤0.001, according to the one-way analysis of variance together with the Newman-Keuls test (n = 4).

We analyzed Akt and p38 MAPK phosphorylation, because both proteins are important mediators downstream of COMP-Ang-1 and are involved in the axon growth and angiogenesis [16], [34]. We show here that COMP-Ang-1 induces phosphorylation of the Akt (Ser 473) and p38MAPK (Thr180/Tyr182) in sciatic nerve of *ob/ob* and *ob/+* mice 60 min after application (Fig. 7). These data support the hypothesis that in sciatic nerves, angio- and neurotrophic- action of COMP-Ang-1 involves phosphorylation of Akt and p38 MAPK upon Tie-2 receptor.

## Discussion

Ang-1, based on its angiogenic properties, has been proposed as a therapeutic strategy to target microvascular diseases in several experimental models. In this line, COMP-Ang-1, a new developed soluble and stabile form of Ang-1, has been shown to prevent the diabetes related retinopathy and nephropathy [35], [36]. Previously, we demonstrated a direct effect of Ang-1 in axonal outgrowth of sensory neurons *in vitro* [13]. These results maybe linked to the recently reported anti-apoptotic and neuritotrophic function of Ang-1 on neurons in CNS [12], [14], [15]. The bifunctional trophic action of Ang-1 both on blood vessels and on nerve fibers prompted us to hypothesize that Ang-1 may have a wider therapeutic range including beneficial effects in neuropathy.

In the present study, we demonstrate that COMP-Ang-1 can reverse the impaired expression of neural structural and gap junction proteins, alteration of endoneural microvessels as well as decreases the infiltration of macrophages and T cells in sciatic nerve of *ob/ob* mice. Additionally, we show that COMP-Ang-1 treatment significantly improves blood glucose and plasma cholesterol concentrations.

A decline of axon calibre, demyelination and impaired neuronal microvasculature belong to the characteristics of PDN [1], [3]. Neurofilaments are the most abundant structural components in axons which determine their calibre and conduction velocities [37]. In streptozotocin-induced diabetes in rats, neuropathy was associated with suppressed mRNA expression of Nfs as well as GAP43 in sensory neurons and their impaired incorporation into distal branches [38]. The decrease in gene expression contributed to inhibition of axonal radial growth and axonal degeneration with consequent reduction of nerve conduction velocity [33], [38]. Our present findings are in accordance with these observations and extent previous findings by demonstrating a markedly decreased expression of Nf68 and GAP43 in sciatic nerve of hyperglycemic *ob/ob* compared with normoglycemic *ob/+* mice. Interestingly, COMP-Ang-1 treatment significantly up-regulates Nf68 and GAP43 protein expressions in sciatic nerve of *ob/ob* mice after 21-day application.

Previously, we have shown that Ang-1 induces the synthesis of Nf68 and the neurite outgrowth through Tie-2 receptor in dorsal root ganglion neurons [13]. Noteworthy, an association between Ang-1/Tie-2 system and the activation of Akt and p38 MAPK pathways was recently reported [39], [40]. The p38 MAPK and Akt belong to recently identified signaling molecules implicated in regeneration of injured nerves [41], [42]. Here, we detect an activation of Tie-2, p38 MAPK and Akt proteins in sciatic nerve upon chronic COMP-Ang-1 treatment. Activation of Akt and p38 MAPK has been associated with morphological responses such as neurite elongation, branching and increase of axon calibre of cultured sensory neurons and PC12 cells as well as of regenerating motor neurons *in vivo* [34], [43], [44]. Therefore, COMP-Ang-1 induced increase of neural structural proteins observed in sciatic nerve of *ob/ob* mice may be mediated through phosphorylation of p38 MAPK and Akt upon Tie-2 receptor. It can not be excluded that these signal cascades are primary activated in DRG neurons and then incorporated into distal fibres. Notably, we have previously shown Ang-1/Tie-2 to cause trans-activation of nerve growth factor tyrosine-kinase receptor A (trkA) in cultivated sensory neurons [13]. Since Akt and p38 MAPK molecules are activated by trkA, interaction between COMP-Ang-1/Tie-2- trkA- Akt signalling pathways are plausible.

Peripheral axons and their associated Schwann cells of endoneurium are isolated from the extracellular space by a diffusion blood–nerve barrier (BNB) also known as the blood-nerve interface. This barrier consists of gap-junctioned perineurial cells of perineurium and endoneurial vascular endothelium [45]. Connexins, expressed by Schwann cells, are an important component implicated in the maintenance of BNB [24]. Altered expression of connexins Cx26, 32 and 43 has been shown to contribute in BNB leakage in diabetic and non-diabetic neuropathy [24]. Furthermore, significant reduction of 26 and 32 Cx isoforms in peripheral nerves of STZ diabetic rats has been reported [4]. In the light of these studies and our results, it seems likely that the markedly decrease of Cx26 and 32 and up-regulation of Cx43 expression or higher number of Iba-1 positive macrophages and CD3 positive T-cells in sciatic nerve of *ob/ob* mice could be closely related to an inflammatory reaction, similar to this observed in degenerated nerve [46].

The lesions with inflammatory infiltrates around epineurial and endoneurial blood vessels and abnormal cytokine production have been shown in various nerve biopsies of patients with diabetic proximal neuropathy [47]. Moreover, we found that the inflammatory cytokine TNFα, mainly expressed in macrophages and Schwann cells, was over expressed in sciatic nerve of *ob/ob* mice compared with normoglycemic controls.

The severity of diabetic neuropathological abnormalities has been related to endoneurial microangiopathy with distinct thickening of basal membrane [31], [48], [49]. Giannini and Dyck [31] have shown that alterations of endoneural microvessels preceed the development of fiber degeneration. In addition the *ob/ob* mice showed impaired density of microvessels with the smallest diameter (<5 µm) compared with ob/+ groups [11]. COMP-Ang-1 enhanced density of endoneural microvessels with smallest diameter in *ob/ob* mice compared to saline controls. Recent studies have shown that microangiopathy is closely associated with disruption of the angiopoietins/Tie-2 system in diabetic mice [19]. We show here that expression of angiopoietin-1 and Tie-2 is significant decreased in sciatic nerve of *ob/ob* mice compared with controls. COMP-Ang-1 treatment caused up-regulation of Ang-1 protein expression and phosphorylation of Tie-2.

*Ob/ob* mice are characterized by obesity and hyperglycaemia [50]. Noteworthy, COMP-Ang-1 improves hyperglycaemia independent of body weight changes. The potential mechanism of COMP-Ang-1 action on improving blood glucose may include vascular enlargement and increased blood flow, subsequently leading to enhanced insulin sensitivity and insulin-stimulated glucose uptake in skeletal muscle [40]. Interestingly, Ade-COMP-Ang-1 decreased plasma glucose without changes in serum insulin level in leptin-receptor deficient diabetic (db/db) mice [36]. The authors have suggested that COMP-Ang-1 has an insulin sensitizing effect in peripheral tissues without direct effect on insulin secretion machinery in pancreatic ß-cells. However, insulin sensitivity and morphology of pancreatic ß-cells were not assessed in this study. Further studies are needed to test whether COMP-Ang-1 treatment may in addition improve insulin sensitivity and/or affect insulin secretion.

Taken together, our data suggest that regenerative changes in sciatic nerve of *ob/ob* mice could be a consequence of: 1) COMP-Ang-1/Tie2 dependent activation of Akt, p38 MAPK signalling pathways in perineurial cells, Schwann cells, pericytes as well as endothelial cells in sciatic nerve and DRG neurons of ob/ob mice; 2) COMP-Ang-1 dependent glucose uptake or a combination of both.

Lack of evident morphological changes of nerve fibers could be explained with the short time of COMP-Ang-1 treatment (21 days) to complete nerve regeneration. In the light of our results, we propose, that decreased inflammation, the increase of nerve structural and gap junction protein expressions as well as growth of endoneural microvessels, are signs of early stages of the peripheral nerve regeneration.

In conlusion, COMP-Ang-1 recovers molecular biomarkers of neuropathy, promotes angiogenesis and suppresses inflammation in sciatic nerves of *ob/ob* mice suggesting COMP-Ang-1 as novel treatment option to improve morphologic and protein expression changes associated with diabetic neuropathy.
